The article "Novel Orthobunyavirus Causing Severe Kidney Disease in Broiler Chickens, Malaysia, 2014–2017" was retracted in 2020. Reason: concerns about the data.

# Novel Orthobunyavirus Causing Severe Kidney Disease in Broiler Chickens, Malaysia, 2014–2017

**DOI:** 10.3201/eid2506.181661

**Published:** 2019-06

**Authors:** Vilmos Palya, Edit Walkóné Kovács, Szilvia Marton, Tímea Tatár-Kis, Balázs Felföldi, Barbara Forró, Marianna Domán, Krisztián Bányai

**Affiliations:** Ceva-Phylaxia Veterinary Biologicals Co. Ltd., Budapest, Hungary (V. Palya, E.W. Kovács, T. Tatár-Kis, B. Felföldi);; Hungarian Academy of Sciences, Budapest (S. Marton, B. Forró, M. Domán, K. Bányai)

**Keywords:** Peribunyaviridae, Orthobunyavirus, Turlock serogroup, Kedah fatal kidney syndrome virus, broiler, chickens, viruses, Malaysia

## Abstract

During 2014–2017, we isolated a novel orthobunyavirus from broiler chickens with severe kidney lesions in the state of Kedah, Malaysia; we named the virus Kedah fatal kidney syndrome virus (KFKSV). Affected chickens became listless and diarrheic before dying suddenly. Necropsies detected pale and swollen kidneys with signs of gout, enlarged and fragile livers, and pale hearts. Experimental infection of broiler chickens with KFKSV reproduced the disease and pathologic conditions observed in the field, fulfilling the Koch’s postulates. Gene sequencing indicated high nucleotide identities between KFKSV isolates (99%) and moderate nucleotide identities with the orthobunyavirus Umbre virus in the large (78%), medium (77%), and small (86%) genomic segments. KFKSV may be pathogenic for other host species, including humans.

In recent years, numerous arboviruses have reportedly caused major outbreaks among domestic or wild birds (*1**,**2*). Most arboviruses associated with widespread epizootics are members of the *Flaviviridae* family, although the poultry industry has been affected by other arboviruses (*3**–**5*). The order *Bunyavirales* comprises at least 9 families and 13 genera. Of the major genera, only viruses of the *Orthobunyavirus*, *Orthohantavirus*, *Orthonairovirus*, and *Phlebovirus* genera infect vertebrates (*6**–**8*). *Orthobunyavirus* is the most diverse genus within the *Bunyavirales* order, comprising ≈170 viruses classified into >18 serogroups on the basis of antigenic relationships; this serology correlates well with the phylogenetic analyses (*9*). For birds, particularly domestic poultry, descriptions of natural infections with orthobunyaviruses are scarce (*10**,**11*). Hubálek et al., in a recent comprehensive review on arboviruses, listed only a few orthobunyaviruses pathogenic to domestic poultry, most likely reflecting a minor role of orthobunyaviruses in poultry diseases (*5*). 

Since 2014, sporadic cases of a new disease in broiler chickens, manifested as clinical signs of lethargy accompanied by some gastrointestinal symptoms and sudden death from severe kidney damage, have been reported in northwestern Malaysia. We identified and characterized the etiologic agent of this disease.

## Materials and Methods

### Detection and Identification of the Etiologic Agent

We collected samples of kidney and cecal tonsils from affected chickens in the field that died and submitted them to the Scientific Support and Investigation Laboratory of Ceva-Phylaxia (Budapest, Hungary) for detection of possible viral agents. The tissue samples were homogenized to give ≈10% (wt/vol) suspension in phosphate-buffered saline pH 7.2. The homogenized samples were centrifuged at 1,000 × *g* for 15 min at 4°C and then filtered through a 0.45-μm membrane. We inoculated 0.2 mL of the filtered supernatant via the chorioallantoic cavity into specific pathogen free (SPF) eggs, 9–11 days old, divided into groups of 5. After inoculation, we checked eggs daily for 7 days and discarded those that died within 24 h. The chorioallantoic fluid was harvested aseptically from embryos that died after 24 h, and these embryos were examined for the presence of gross pathologic lesions. If at the end of the 7-day observation period no embryos had died, we removed the eggs with live embryos and kept them at 4°C for 24 h and then collected the chorioallantoic fluid for the next passage. We conducted 3 blind passages before considering a sample negative for pathogens.

The chorioallantoic fluid of the embryos showing pathologic lesions was inoculated onto LMH (chicken hepatocellular carcinoma) and Vero (African green monkey kidney) cell cultures and checked for cytopathogenic agents. LMH cells were also used for propagation and titration of the isolated virus and for reisolation of the virus from kidney samples from experimentally infected chickens.

Supernatants of tissue cultures showing cytopathologic changes were centrifuged at 10,000 × *g* for 5 min, and 200 μL of the supernatant was used for nucleic acid extraction by use of the ZiXpress32 Viral Nucleic Acid Extraction Kit and ZiXpress32 robot (Zinexts Life Science, http://www.Zinexts.com). Random primed reverse-transcription PCR (RT-PCR) was performed as described elsewhere (*12**,**13*). We subjected 100 ng of cDNA to enzymatic fragmentation and adaptor ligation, following the manufacturer’s recommendations (NEBNext Fast DNA Fragmentation & Library Prep Set for Ion Torrent; New England Biolabs, https://www.neb.com). The resulting cDNA libraries were measured on Qubit 2.0 equipment by using the Qubit dsDNA BR Assay kit (Invitrogen, https://www.thermofisher.com). The isothermal emulsion PCR that produced clonally amplified libraries was conducted according to the manufacturer’s protocol by using the IA 500 kit (Life Technologies, https://www.thermofisher.com). Enrichment of the templated beads (on an Ion OneTouch ES machine; Life Technologies) and further steps of presequencing setup were performed according to the manufacturer’s 200-bp protocol. We strictly followed the sequencing protocol recommended for the Ion PGM Hi-Q View Sequencing Kit on a 316 v2 chip (Life Technologies).

Sanger sequencing was used to validate results obtained by the viral metagenomics approach. Primer pairs were designed to amplify 0.8–1.2-kb fragments (not shown). The BrightDye Terminator Cycle Sequencing Kit (NimaGen, https://www.nimagen.com) was used in the amplification reaction, and dye-labeled products were run on an ABI 3500 sequencer (Life Technologies).

Sequence reads obtained by next-generation sequencing were trimmed by using CLC Genomics Workbench version 7 (http://www.clcbio.com). The minimal read length parameter was set to 40. The same software was used to assemble the genome sequence. After visually inspecting the sequence mappings, we created 1 consensus sequence for all 3 genome segments (small [S], medium [M], and large [L]). Sanger sequencing outputs were analyzed by using BioEdit software (*14*). Sequence contigs from the 2 sequencing platforms were assembled and further edited by using GeneDoc (*15*) and BioEdit software and then analyzed by similarity search with BLAST (*14**–**16*). We deposited newly generated nucleotide sequences into GenBank (accession nos. MK047401–MK047415). Multiple alignments were prepared by using the TranslatorX online program (*17*) and manually adjusted in GeneDoc, whereas phylogenetic analysis by the maximum-likelihood and the neighbor-joining methods was performed by using MEGA6 software (*18*). The coding potential was predicted by using ORF Finder (http://www.ncbi.nlm.nih.gov/gorf/gorf.html).

### Development of Diagnostic RT-PCR

For assay development and quantification of the novel orthobunyavirus genomic RNA in organ samples of the experimental animals, we extracted viral RNA as previously described and designed primers and probes for the S genomic segment of the novel orthobunyavirus. The reaction mixture of quantitative RT-PCR (qRT-PCR) that we used was composed of 10 μL 2× qPCRBIO Probe 1-Step Mix (PCR Biosystems, http://www.pcrbio.com), 1.6 μL S gene specific forward (5′ GGGTAGCACTAGCATTTATCCA 3′) and reverse (5′ TGTAGACACCCACAAACGTATC 3′) primers (each from 10 μM stock solutions), 0.5 μL S gene specific probe (5′ [FAM] AGCTCACATACGAGGATACACAGGA [BHQ] 3′) from a 10 μM stock solution, 1 μL 20X RTase with RNase inhibitor, 0.3 μL nuclease-free water, and 5 μL RNA. The thermal profile of the qRT-PCR was as follows: reverse transcription at 50°C for 10 min terminated by heating to 95 °C for 2 min, followed by amplification performed in 40 cycles consisting of denaturation at 95°C for 5 s and hybridization and elongation at 60°C for 20 s. Throughout the study, we used a Mic qPCR cycler (Bio Molecular Systems, https://biomolecularsystems.com), kindly provided for the project by Péter Kisfali, Amplicon Ltd.).

To test the assay specificity, we used a number of viruses from our strain collection, including avian nephritis virus (*Astroviridae*); QX-like, 4/91-like, and Massachusetts-like infectious bronchitis virus strains (*Coronaviridae*); representative isolates of avian metapneumovirus A, B, and C and Newcastle disease virus (*Paramyxoviridae*); isolates of influenza (H9N2) and (H5N8) viruses (*Orthomyxoviridae*); and Tembusu virus (*Flaviviridae*).

### Experimental Reproduction of the Disease

We tested the pathogenicity of 1 of the isolates (D2756/1/2014/MY) in 5-day-old broiler chickens purchased from a commercial hatchery in Hungary. We inoculated 10 chickens with 0.2 mL of 5.1 log_10_ 50% tissue culture infective dose (TCID_50_) of the isolate by either the subcutaneous or oral route; for negative controls, we inoculated 5 chickens of the same age with phosphate-buffered saline pH 7.2. We kept all birds in isolators with negative pressure and monitored them daily for overt clinical signs and death for 26 days after inoculation.

We recorded gross lesions of birds that died during the 26-day postinoculation period and collected samples from the spleen, liver, kidney, heart, pancreas, small intestine, bursa, and thymus and placed them in 10% buffered formalin for histologic analysis. We also collected tissue samples (spleen, liver, kidney, heart, intestine, and bursa) from 5 chickens in the subcutaneously infected group and 4 chickens from the orally infected group that died and processed them for viral RNA detection by using qRT-PCR. We euthanized all remaining birds and inspected them for gross pathologic lesions, collecting samples for histologic analysis (spleens, livers, kidneys, hearts, and bursa Fabricii) and qRT-PCR (spleens and kidneys from all; hearts, livers, bursa Fabricii, and cecal tonsils from a few).

### Histologic Analyses

Tissue samples were processed according to standard histologic procedures. Samples were embedded in paraffin, cut in 5-μm sections, stained with hematoxylin and eosin or trichrome, and examined under light microscopy.

## Results

### Epidemiologic and Clinical Observations

The first outbreaks of the disease occurred during July–September 2014 and recurred during the same months each subsequent year. All cases were from broiler farms with open-sided houses in Kedah (Figure 1).

**Figure 1:** Locations of cases of severe kidney disease in broiler chickens, Malaysia, 2014–2017. Black icons indicate locations of investigated outbreaks. Colored boxes indicate road numbers. Inset indicates area affected by outbreaks within Malaysia.

Several chickens in the affected flocks became listless and exhibited signs of diarrhea. Affected birds died soon after the appearance of the first clinical signs. The disease sometimes occurred in birds ≈1 week of age but more routinely in those 2–4 weeks of age. Mortality rates varied within a wide range, from a low percentage to 30%–40% (Figure 2). 

**Figure 2:** Daily mortality rates among broiler chickens with severe kidney disease, Malaysia, 2014–2017. A) Flock affected by the 2014 outbreak. B) Four flocks affected by the 2017 outbreaks.

The most striking lesions in dead chickens were pale, swollen kidneys with uric acid deposits, frequently localized in the tubules and ureters (Figure 3) and also found on the surface of serosa covering the visceral organs. The livers were moderately enlarged and fragile. The heart muscle was pale. No obvious gross lesions were seen in any other organs.

**Figure 3:** Gross pathologic appearance of kidney from a chicken with severe kidney disease naturally infected with a novel orthobunyavirus (Kedah fatal kidney syndrome virus), Malaysia, 2014–2017.

### Etiologic Agent

From the kidney and cecal tonsil samples submitted from 1 affected chicken in 2014 and 3 affected chickens in 2017, we obtained 5 virus isolates after 1 blind passage in SPF embryos. Embryo deaths occurred 3–5 days after inoculation with the organ homogenates. The dead embryos exhibited severe subcutaneous edema, congestion, and hemorrhages on the skin. No hemagglutinating agents were observed when chicken red blood cells were used in analysis of allantoic fluid from dead embryos.

Cytopathic effect was evident at 48–72 hours after inoculation of LMH and Vero cell cultures with the allantoic fluid from dead embryos. Elongated or rounded dark cells were seen in irregular clusters, expanding very fast to affect the whole cell sheet within 24–36 hours. The virus grown on LMH cell cultures reached a titer of 6.3–6.5 log_10_ TCID_50_/mL.

Viral metagenomics performed from 2 cell culture supernatants (D2756/1/2014/MY and D2756/2/2014/MY) identified sequence scaffolds with greatest BLAST hits to the orthobunyavirus Umbre virus (Turlock serogroup). The most 3′ and 5′ ends of the genomic RNA could not be determined with this method. To confirm the sequencing results obtained by next-generation sequencing, we also performed Sanger sequencing. The obtained nearly full-length genome sequences (L segment ≈6.9 kbp, M segment ≈4.3 kbp, S segment ≈0.8 kbp) showed >99% nt sequence identities between isolates D2756/1/2014/MY and D2756/2/2014/MY. When we compared sequences with Umbre virus, we identified 78% nt sequence identities along L, 77% along M, and 86% along S genomic segments.

### Diagnostic qRT-PCR

The S genomic segment contained an ≈200-bp fragment that shared high sequence homology with Umbre virus. Primers and probes had been designed to detect Malaysia orthobunyavirus isolates and Umbre virus, although the assay was not tested against Umbre virus or other closely related strains within the Turlock serogroup. The assay exhibited high specificity when tested against a variety of viruses characterized by kidney tropism and was able to reproducibly detect the viral RNA from tissues that corresponded to as few as 3 TCID_50_/mL virus culture supernatant (or 0.03 TCID_50_ virus/5 μL RNA). The kidney samples submitted from the sick poultry in the field during 2014 and 2017 contained RNA copies corresponding to a viral titer of 9.00 × 10^4^ to 4.81 × 10^5^ TCID_50_ of infectious virus per gram of organ specimen. Phylogenetic analysis based on the partial amino acid sequences of proteins encoded by the L, M, and S segments showed that all 5 isolates detected from 4 different outbreak cases over a 3-year period were highly similar in the regions analyzed (Figure 4).

**Figure 4:** Phylogenetic trees of novel orthobunyavirus (Kedah fatal kidney syndrome virus) identified as the cause of severe kidney disease, Malaysia, 2014–2017 (black diamonds) and reference orthobunyaviruses. A) Large genome segment tree; B) medium gene–derived tree; C) small genome segment derived tree. Scale bars indicate nucleotide substitutions per site.

### Experimental Reproduction of the Disease

The pathologic condition of chickens in the field could be reproduced by experimental infection of chickens with 1 of the selected isolates (D2756/1/2014/MY). From postinoculation day 3, chickens became listless and showed loss of appetite. Deaths occurred during postinoculation days 3–5 in the subcutaneously infected group and started 2 days later (postinoculation day 5) in the orally infected group. The mortality rate was higher for the group infected by the subcutaneous route (Figure 5).

**Figure 5:** Daily survival rates among chickens experimentally infected with a novel orthobunyavirus (Kedah fatal kidney syndrome virus), isolated from broiler chickens with severe kidney disease, Malaysia, 2014–2017.

After clinical signs appeared, the chickens died within 12–24 hours. In those that died, gross lesions were mainly confined to the kidneys, which were pale and swollen with distended ureters filled with uric acid (Figure 6, panel A). In some chickens, visceral gout also developed (Figure 6, panel B). Other gross lesions that could be observed in most dead chickens were accumulation of serous exudate in the abdominal cavity and pericardium, signs of liver degeneration, and discoloration of the heart muscle. The chickens in the control group remained healthy throughout the observation period.

**Figure 6:** Gross pathologic appearance of chickens experimentally infected with a novel orthobunyavirus (Kedah fatal kidney syndrome virus) isolated from chickens with severe kidney disease, Malaysia, 2014–2017. A) Swollen and pale kidney; B) uric acid crystals on viscera (gout).

### Histopathologic Findings

In the organs collected from the experimentally infected chickens that died, the predominant histologic lesions were in the kidney, liver, heart, and lymphoid organs. The most consistent lesions were tubulonephrosis with occasional tubular epithelium necrosis; intraglomerular urolithiasis and multifocal interstitial lympho-histiocytic infiltration (Figure 7, panel A); vacuolic degeneration and disintegration of liver cells with signs of hepatitis (Figure 7, panel B); acute serous myocarditis; and depletion of lymphocytes with scattered lymphocyte necrosis in the lymphoid organs (spleen, bursa Fabricii, and thymus) (Figure 7, panels C and D).

**Figure 7:** Histologic appearance of lesions in tissues from chickens experimentally infected with a novel orthobunyavirus (Kedah fatal kidney syndrome virus) isolated from broiler chickens with severe kidney disease, Malaysia, 2014–2017. A) Kidney, showing urate deposits in the dilated Bowman’s capsule (arrows) and degeneration and dilatation of proximal convoluted tubules. Trichcrome stain; original magnification ×200. B) Liver, showing vacuolar degeneration of hepatocytes and disorganization of lobular structure. Hematoxylin and eosin (H&E) stain; original magnification ×400. C) Spleen, showing marked lymphoid depletion and lymphocyte necrosis in the Malpighian body and vacuolation of reticulocytes in the red pulp (arrow). H&E stain; original magnification ×400. D) Bursa Fabricii, showing atrophy of bursal follicles with marked lymphoid depletion in the medullary region (arrow). H&E stain; original magnification ×200.

Histopathologic changes were nearly completely missing in the birds sampled at the end of the experiment. Only some focal interstitial nephritis, hepatitis, and myocarditis could be found in a few birds.

### Viral RNA in Tissue Samples from Infected Chickens

High viral loads in the different organ samples of dead chickens were similar, irrespective of the route of infection and time of death (Table). These results suggest that the virus could cause a high level of viremia and could replicate at a significant level in different organs (different cell types). The virus-specific nucleic acid was still present in the spleen of healthy chickens at the end of the observation period, but no viral RNA could be detected in kidney, cecal tonsil, and bursa tissues from these chickens.

**Table:** Viral load in organs of chickens inoculated with orthobunyavirus isolated from broiler chickens with severe kidney disease, Malaysia, 2014*

Inoculation type and date of death, dpi	Viral load, log10 TCID50/g					
	Spleen	Kidney	Heart	Liver	Cecal tonsil/intestine	Bursa
Subcutaneous						
4	5.8	5.1	NS	NS	NS	NS
5	4.7	5.9	NS	NS	NS	NS
5	4.1	5.7	NS	NS	NS	NS
5	5.3	5.4	NS	NS	NS	NS
6	5.1	5.4	NS	NS	NS	NS
Oral						
5	5.6	6.5	NS	NS	NS	NS
5	5.9	5.8	5.7	4.3	6.3	4.7
6	5.6	6.2	NS	NS	NS	NS
6	5.4	6.8	5.5	4.2	5.6	4.4
26	4.2	Neg	NS	NS	Neg	Neg
26	4.7	Neg	NS	NS	Neg	Neg
26	4.4	Neg	NS	NS	Neg	Neg

*dpi, days postinfection; neg, negative; NS, not sampled; TCID50, 50% tissue culture infective dose.

## Discussion

We found the causative agent of the disease outbreak of severe kidney damage among broiler chickens in Malaysia in 2014 to be a newly emerging orthobunyavirus. On the basis of the main pathologic features of the disease seen in the field and after experimental infection, we propose that the virus be designated Kedah fatal kidney syndrome virus (KFKSV) of broilers.

Analysis of the near full-genome sequence of 2 isolates, D2756/1/2014/MY and D2756/2/2014/MY, demonstrated that the virus is similar to Umbre virus, which belongs to the Turlock serogroup of the *Orthobunyavirus* genus (*19*). This serogroup is represented by 2 species and several virus isolates detected in Africa, Asia, Europe, and the Americas (*20*). So far, little information has been collected about the pathogenic potential of viruses belonging to the Turlock serogroup. Antibody response and transient viremia have been observed in chickens experimentally infected with Turlock virus (*21*).

Umbre virus was isolated during the 1950s from *Culex* mosquitoes and birds (*22*,*23*) from India and Malaysia, and antibodies have been measured in serum of wild birds and sentinel chickens from Malaysia (*24*). Although D2756/1/2014/MY, which we isolated, is genetically related to Umbre virus, we propose the name Kedah fatal kidney syndrome virus of broilers on the basis of its unique pathologic characteristics in meat-type chickens.

Several viruses within the *Orthobunyavirus* genus are of major veterinary and public health concern (*5*). Because KFKSV is a newly emerging virus, no experimental data are available regarding its pathogenicity and transmissibility. Disease in chickens could be reproduced by oral infection even though most orthobunyaviruses are vectorborne and the field cases in Malaysia occurred during mosquito season. Our results show that, after oral infection, high levels of virus could be detected in internal organs (including intestines) of infected chickens, which suggests that direct bird-to-bird transmission may contribute to the spread of this virus within an infected flock. The disease characteristics (e.g., sudden outbreaks, fast spread, and high morbidity rates) further support the existence of direct bird-to-bird transmission within a flock; however, the role of arthropods in introducing infection into a flock cannot be ruled out because of the seasonal occurrence of the disease. The fast spread of the disease in a flock and our experimental infection results, which proved that infection by the oral route is efficient, strongly suggest that mosquitoes may not be the exclusive vehicle for transmission of this virus within a flock.

The D2756/1/2014/MY isolate of KFKSV was highly pathogenic in young broiler chickens, causing mortality rates of 50%–70% and severe gross and histopathologic lesions in the kidneys and liver after experimental infection. The gross and histopathologic changes caused by the isolate were similar to those found in field-infected chickens. The virus could be detected from all tested internal organs of dead chickens, including intestines, but the spleen samples collected from asymptomatic chickens after recovery were also positive for KFKSV 3 weeks after infection. Therefore, investigation of virus persistence and transmission is needed.

There are no commercially available or standardized tests for diagnosing bunyavirus infections in poultry. Establishing a diagnosis requires submitting samples to specialized reference laboratories. KFKSV can be isolated and grown in chicken embryos and can be propagated in LMH and Vero cells. When reported disease and clinical history of a flock includes kidney lesions, diagnostic laboratories can use the molecular diagnostic method we describe in this article to check submitted materials for this newly discovered emerging species of orthobunyavirus. Similar kidney lesions could be observed after infection with avian infectious bronchitis virus, astrovirus, and leucocytozoonosis. Diagnosis of these infections is generally based on detection by RT-PCR and sequencing, virus isolation, and demonstration of an immune response by virus neutralization or enzyme immunoassay.

For determining a possible viral origin of an idiopathic disease, the viral metagenomics technique is useful, as is demonstrated by our discovery of this novel orthobunyavirus. The potential of this virus to spread to other animal species or humans cannot be excluded. Therefore, studies in which additional data are collected to elucidate the pathogenic potential of this virus in avian and other animal species should be initiated. Studies to scrutinize its potential as a public health hazard should also be considered. Because of the zoonotic nature of some orthobunyaviruses closely related to KFKSV (*5*,*25*–*27*), we highlight the need for wider surveillance of KFKSV in birds and mammals of other species in a more extended geographic area. Research in the surveillance of putative disease vectors and the possible prevalence of this virus in livestock and wildlife should be encouraged. The molecular diagnostic assay that we developed could help these research and disease surveillance efforts in the affected area, although the extent of its applicability against a broader diversity of orthobunyaviruses needs to be validated.

## References

[1] Pello SJ, Olsen GH. Emerging and reemerging diseases of avian wildlife. Vet Clin North Am Exot Anim Pract. 2013;16:357–81. 10.1016/j.cvex.2013.02.00123642867

[2] Chan JF-W, To KK-W, Chen H, Yuen K-Y. Cross-species transmission and emergence of novel viruses from birds. Curr Opin Virol. 2015;10:63–9. 10.1016/j.coviro.2015.01.00625644327PMC7102742

[3] Liu P, Lu H, Li S, Wu Y, Gao GF, Su J. Duck egg drop syndrome virus: an emerging Tembusu-related flavivirus in China. Sci China Life Sci. 2013;56:701–10. 10.1007/s11427-013-4515-z23917842

[4] Cadar D, Lühken R, van der Jeugd H, Garigliany M, Ziegler U, Keller M, et al. Widespread activity of multiple lineages of Usutu virus, western Europe, 2016. Euro Surveill. 2017;22:30452. 10.2807/1560-7917.ES.2017.22.4.3045228181903PMC5388094

[5] Hubálek Z, Rudolf I, Nowotny N. Arboviruses pathogenic for domestic and wild animals. Adv Virus Res. 2014;89:201–75. 10.1016/B978-0-12-800172-1.00005-724751197

[6] Horne KM, Vanlandingham DL. Bunyavirus-vector interactions. Viruses. 2014;6:4373–97. 10.3390/v611437325402172PMC4246228

[7] Elliott RM. Bunyaviridae. In: Knipe DM, Howley PM, editors. Fields virology, 6th ed, vol. 1. Philadelphia: Wolters Kluwer Health; 2013. p. 1244–82.

[8] International Committee on Taxonomy of Viruses. Master species list 2017 v1.0 [cited 2018 Mar 12]. https://talk.ictvonline.org/files/master-species-lists

[9] Wilson WC, Gaudreault NN, Hossain MM, McVey DS. Lesser-known bunyavirus infections. Rev Sci Tech. 2015;34:419–29. 10.20506/rst.34.2.236826601445

[10] Whitmer SLM, Yadav PD, Sarkale P, Chaubal GY, Francis A, Klena J, et al. Characterization of unknown orthobunya-like viruses from India. Viruses. 2018;10:E451. 10.3390/v1009045130149496PMC6165560

[11] Al’kovskhovskiĭ SV, Shchetinin AM, L’vov DK, Shchelkanov MI, Deriabin PG, L’vov DN, et al. [The Khurdun virus (KHURV): a new representative of the orthobunyavirus (Bunyaviridae)]. Vopr Virusol. 2013;58:10–3.24354059

[12] Djikeng A, Halpin R, Kuzmickas R, Depasse J, Feldblyum J, Sengamalay N, et al. Viral genome sequencing by random priming methods. BMC Genomics. 2008;9:5. 10.1186/1471-2164-9-518179705PMC2254600

[13] Bányai K, Kemenesi G, Budinski I, Földes F, Zana B, Marton S, et al. Candidate new rotavirus species in Schreiber’s bats, Serbia. Infect Genet Evol. 2017;48:19–26. 10.1016/j.meegid.2016.12.00227932285PMC7106153

[14] Hall TA. BioEdit: a user-friendly biological sequence alignment editor and analysis program for windows 95/98/NT [cited 2018 Oct 4]. http://jwbrown.mbio.ncsu.edu/JWB/papers/1999Hall1.pdf.

[15] Nicholas KB, Nicholas HB Jr, Deerfield DWII. GeneDoc: analysis and visualization of genetic variation. Embnew News. 1997;4:14.

[16] Altschul SF, Gish W, Miller W, Myers EW, Lipman DJ. Basic local alignment search tool. J Mol Biol. 1990;215:403–10. 10.1016/S0022-2836(05)80360-22231712

[17] Abascal F, Zardoya R, Telford MJ. TranslatorX: multiple alignment of nucleotide sequences guided by amino acid translations. Nucleic Acids Res. 2010;38(suppl_2):W7–13. 10.1093/nar/gkq291PMC289617320435676

[18] Tamura K, Stecher G, Peterson D, Filipski A, Kumar S. MEGA6: molecular evolutionary genetics analysis version 6.0. Mol Biol Evol. 2013;30:2725–9. 10.1093/molbev/mst19724132122PMC3840312

[19] Calisher CH, Lazuick JS, Wolff KL, Muth DJ. Antigenic relationships among Turlock serogroup Bunyaviruses as determined by neutralization tests. Acta Virol. 1984;28:148–51.6203387

[20] Shchetinin AM, Lvov DK, Deriabin PG, Botikov AG, Gitelman AK, Kuhn JH, et al. Genetic and Phylogenetic Characterization of Tataguine and Witwatersrand Viruses and Other Orthobunyaviruses of the Anopheles A, Capim, Guamá, Koongol, Mapputta, Tete, and Turlock Serogroups. Viruses. 2015;7:5987–6008. 10.3390/v711291826610546PMC4664991

[21] Scott TW, McLean RG, Francy DB, Mitchell CJ, Card CS. Experimental infections of birds with Turlock virus. J Wildl Dis. 1983;19:82–5. 10.7589/0090-3558-19.2.826411942

[22] Yadav PD, Mishra AC, Mourya DT. Molecular characterization of Umbre virus (*Bunyaviridae*). Virol J. 2008;5:115. 10.1186/1743-422X-5-11518842123PMC2586634

[23] Dandawate CN, Rajagopalan PK, Pavri KM, Work TH. Virus isolations from mosquitoes collected in North Arcot district, Madras state, and Chittoor district, Andhra Pradesh between November 1955 and October 1957. Indian J Med Res. 1969;57:1420–6.4395257

[24] Wallace HG, Rudnick A, Rajagopal V. Activity of Tembusu and Umbre viruses in a Malaysian community: mosquito studies. Mosq News. 1977;37:35–42.

[25] Sakkas H, Bozidis P, Franks A, Papadopoulou C. Oropouche fever: a review. Viruses. 2018;10:E175. 10.3390/v1004017529617280PMC5923469

[26] Noronha LE, Wilson WC. Comparison of two zoonotic viruses from the order Bunyavirales. Curr Opin Virol. 2017;27:36–41. 10.1016/j.coviro.2017.10.00729128744

[27] Lundström JO. Mosquito-borne viruses in western Europe: a review. J Vector Ecol. 1999;24:1–39.10436876

